The article "Evolutionary Analysis of Supply Chain Integration Strategy on Chinese Steel-Producing Firms considering Policy Risk Cost Factor" was retracted in 2023. Reasons: unreliable results or conclusions; concerns about the data; concerns about the results or conclusions; concerns about the peer review.

# Evolutionary Analysis of Supply Chain Integration Strategy on Chinese Steel-Producing Firms considering Policy Risk Cost Factor

**DOI:** 10.1155/2022/1136601

**Published:** 2022-06-25

**Authors:** Lequn Zhu, Ran Zhou, Xiaojun Li, Jie Chen

**Affiliations:** ^1^Tianjin Research Institute for Water Transport Engineering, M.O.T., Tianjin, China; ^2^Department of Management, Shenzhen Polytechnic, Shenzhen, China

## Abstract

Despite a number of adverse factors, China's steel industry has maintained a rapid growth trend. China continues to consume two-thirds of the world's iron ore, the majority of which is imported. In this context, Chinese steel companies have begun to consider integrating their supply chains to increase efficiency and lower costs. However, the increasingly volatile international environment makes this an extremely risky proposition. As a result, the issue of how Chinese steel producers should participate in global supply chain integration has emerged as a critical research question that requires investigation. In this paper, we examine the supply chain integration problem using a typical China–Australia steel trade as an example. Specifically, we discuss in detail whether relevant firms should continue to promote supply chain integration in the Chinese–Australian steel industry, as well as the decision boundary of influence, using evolutionary game theory and policy risk cost factors. The empirical analysis demonstrates that policy risk has a range of effects on different types of steel firms. Even when international tensions are considered, smaller steel companies may retain a greater willingness to integrate their supply chains. Overall, the above findings can provide necessary decision support for enterprises to formulate supply chain management strategies.

## 1. Introduction

Iron ore is one of the main raw materials of the steel industry. The bulk of Chinese iron ore reserves is of a poor grade, technically difficult to exploit, and located far from the major steel-producing centers on the eastern seaboard [1] (pp. 1084–1094). With the rapid development of the domestic steel industry, Chinese iron ore reserves and their exploitation cannot meet the large demand. Australia has long been China's primary iron ore supplier [2] (pp. 95–106). Despite the impact of the COVID-19 pandemic in 2019 and the deterioration of China–Australia relations, the two countries' iron ore trade has remained relatively stable. In 2020, China imported 712.986 million tons of iron ore from Australia (see Figure 1), accounting for 60.93 percent of total Chinese iron ore imports. It demonstrates that Australia remains a vital and irreplaceable source of high-quality iron ore for China.

Of course, the impact of political factors on the China–Australia iron ore trade cannot be underestimated. With the development of an intense rivalry between the two countries, both governments have imposed a number of explicit and implicit restrictions on iron ore trade and business cooperation in related areas. The Chinese government, for example, has restricted the offloading of iron ore ships from Australia and is actively developing or seeking alternative sources of Australian iron ore in Southeast Asia. The Australian government also announced plans to cancel mining rights already acquired by some Chinese companies in April 2021. Once implemented, the aforementioned measures will undoubtedly result in massive financial losses for the affected companies.

Although political factors have had a significant negative impact on the two countries' iron ore trade, both governments are well aware of the economic fundamentals: the iron ore trade between Australia and China cannot be artificially halted [3] (pp. 331–339). On the one hand, the China–Australia iron ore trade is critical to Australia's economic development, and a complete shutdown of the China–Australia iron ore trade would severely impair Australia's economic growth. On the other hand, China would have difficulty obtaining such a large supply of high-quality iron ore from other global suppliers. Additionally, Chinese companies have already invested significant capital in Australia. Numerous projects have been secured or put into operation, and the industrial integration of related resources is progressing steadily. As a result, we believe that with the adjustment of the new U.S. administration's anti-China sanctions policy, the intensity of trade frictions between China and Australia is likely to decrease, resulting in the recovery of the China–Australia iron ore trade.

In the aforementioned complex international political and economic environment, how Chinese steel producers should participate in the Chinese–Australian steel industry's supply chain integration (SCI) has become an important issue worth investigating. SCI takes many forms in practice, including the purchase of mining rights, direct investment in ore exploration or smelting, and so forth. Although SCI can help steel producers lower their operating costs and improve their competitiveness, it can also make them more vulnerable to changes in the trade environment and policies, exposing them to more operational risks. As a result, the decision makers in Chinese steel producers and the Chinese government must respond two questions in the face of an increasingly complex economic and trade environment, which are as follows: is it necessary for steel producers to continue to promote SCI? What effect will trade restrictions on iron ore have on Chinese steel producers' SCI? Based on evolutionary game theory, we will discuss these research questions in depth in this paper.

Overall, the contributions of this paper are broadly twofold. Firstly, for the first time, we consider the impact of political factors on related trade activities in the discussion of iron ore trade. Secondly, we use an evolutionary game model to provide decision recommendations of practical value for Chinese steel firms' decisions.

The remainder of this paper is divided into the following sections: Section 2 examines the relevant literature and identifies the research gap this paper attempts to fill. The model is introduced in Section 4, where we also analyze the evolutionary game and the case study we later conduct in Section 5.  Section 3 introduces the evolutionary game framework of this paper, introducing the relevant hypotheses and the game mechanism. Section 4 introduces the model, where we also analyze the evolutionary game, and Section 5 introduces the case study we conduct. Finally, Section 6 contains the paper's conclusion and policy recommendations.

## 2. Literature Review

Over the years, scholars' focus on SCI practices has shifted significantly [4] (pp. 353–361) [5] (pp. 42–55). The majority of these studies agree on the fundamental premise that implementing SCI effectively throughout the supply chain is vital to modern businesses' capacity to maintain a competitive edge [6] (pp. 24–41).

Robinson believes that a paradigm shift is taking place in which value is sought and delivered through integrative efficiency rather than operational efficiency [7] (pp. 89–106). Effective SCI is crucial for some firms to minimize supply chain expenses and achieve a competitive edge [8] (pp. 119–134). Establishing strategic partnerships or alliances with suppliers increases the interaction between businesses and suppliers, enhancing the supply chain's performance [9] (pp. 58–71). SCI appears to be a primary method for Chinese steel makers to address their iron ore supply chain difficulties. For example, Baosteel Group, the second largest steel-producing company in China and the fourth largest steel-producing company in the world, established Baosteel Resources as a wholly owned subsidiary that is mainly engaged in mineral resource investment, trade, and logistics services and claimed that its 2009 investment in Aquila Resources would strengthen Baosteel's control over resources and lower purchasing costs.

Although most researchers accept that SCI can contribute to increasing supply network performance, it is notable that only a few studies have focused on the conditions of implementing SCI because SCI is not applicable in all cases. Mouritsen et al. demonstrate that similar levels of implementation of SCI practices do not always result in comparable improvements [10] (pp. 686–695). O'Leary-Kelly and Flores, as well as Wong et al., emphasize the urgent need to understand the conditions that maximize performance improvements [11] (pp. 221–240) [12] (pp. 604–615). Smith et al. note that trade costs along domestic and international supply chains in Asian economies can be significantly reduced by improving the logistics performance in each mode of transport involved in various logistics and supply chain transactions [13].

If steel-producing firms choose SCI, they must bear a considerable investment cost and substantial financial pressure. Although Chinese steel-producing firms can obtain assistance from the Chinese state-owned banking system, which can provide steel-producing firms loan finance on concessionary terms for investment in iron ore projects overseas, applying this strategy entails high risk and capital costs. Therefore, it is essential to investigate the conditions under which SCI can be more beneficial for Chinese steel-producing firms. As a result, it is critical to investigate the circumstances under which SCI can be more beneficial to Chinese steel producers.

Numerous scholars have already conducted research on the implementation conditions of SCI. According to Beresford et al., the optimal mode of transport for iron ore is a combination of sea and rail [14] (pp. 32–42). The global supply chain for iron ore is complex and involves multiple, diverse stakeholders, including foreign iron ore suppliers, foreign port authorities, shipping companies, domestic port authorities, and domestic logistics service providers. This makes it extremely difficult to directly assess SCI implementation conditions. However, the steel production market is typically monopolistic, which allows for the possibility of analyzing the implementation of SCI in this market. For instance, a monopolistic steel manufacturer can have a significant impact on another firm's decision to adopt SCI by adjusting the price of its products.

This study builds on this foundation by employing an evolutionary game approach to analyze the decision-making behavior of participants in the steel-producing market. From a managerial perspective, this paper emphasizes the critical nature of comprehending the conditions that enable SCI to be highly effective, as well as the impact of government relationships on the revenue of the companies involved and their willingness to integrate the supply chain.

## 3. Game Model

### 3.1. Problem Description and Setting

As the systematic establishment of SCI is not easily accomplished in a short period of time [5] (pp. 42–55), we can regard SCI as a long-term process. Additionally, while implementing SCI may result in increased productivity, it may also amplify the impact of political risk factors on a company's manufacturing activities. Because SCI connects steel producers to iron ore suppliers, the more integrated a supply chain, the greater the political risk the businesses face. We established the steel and iron ore supply markets as follows based on the foregoing facts.

Assume there are two distinct types of firms in the market (designated firm A and firm B), and they differ substantially in terms of not only profitability but also in SCI costs [15] (pp. 235–253). For each type of firm, two pure strategies are assumed: SCI or no SCI, and to simplify the problem, SCI is defined as the acquisition of mineral resource exploration rights, resource extraction facilities, and transportation investments. Additionally, we assume that the two types of firms are in an incomplete information game relationship, which means that they both have limited cognition and lack access to all necessary information when making SCI decisions. As a result, they cannot make perfectly rational decisions and must instead revise their decision strategies based on incomplete information, gradually improving their position in the game through adaptive learning in the process of continuous improvement. Furthermore, we postulate that the outcomes of the SCI decisions made by two distinct types of firms can affect one another.

The cost of SCI is assumed to consist of two components [16] (pp. 281–294). One is the fixed cost incurred as a result of chain integration, which includes investment in resource exploration, excavation, and transportation. The other is the loss incurred as a result of investment not being recovered (or the project being unable to proceed) because of political factors when Chinese firms invest their fixed assets overseas. In the following, we will utilize the fixed asset investment loss ratio to quantify the cost increase caused by political considerations. For instance, if we assume that the relationship between the Chinese and Australian governments deteriorates significantly and Chinese firms' licenses to develop mineral resources in Australia are completely terminated, then the associated loss ratio of investment is 100 percent, and this coefficient is treated as an exogenous variable in subsequent discussions.

In summary, we assume that the firms A and B face limited cognitive and information access difficulties, are not completely rational, and have asymmetric strategy choices and benefits. As a result, the problem is an asymmetric evolutionary game with imperfect information. As firms A and B must determine whether to integrate their supply chains in this game, there are four possible outcomes, as illustrated in Figure 2. We use the vectors (*π*_*A*_^1^, *π*_*B*_^1^), (*π*_*A*_^2^, *π*_*B*_^2^),  (*π*_*A*_^3^, *π*_*B*_^3^), and (*π*_*A*_^4^, *π*_*B*_^4^) to denote the payoff of each game participant in different situations. For instance, in the first case, *π*_*A*_^1^ symbolizes the payment to firm A (where firms A and B implement integration strategies). The payouts of firms A and B are calculated in Table 1 for a variety of game outcomes.

### 3.2. Evolutionary Game Model

We investigate the behavior of firms A and B described above in this paper using an evolutionary game framework. The fundamental premise of this framework is to represent the two distinct types of firms as two distinct biological groups, dubbed group A and group B [17] (pp. 32–38). Individuals in the two groups mimic and refine their own strategies based on the available local information, and therefore, they learn to optimize their returns adaptively in a multistage (denoted as t) dynamic game process. Finally, the two groups' game results are evaluated in terms of the proportion of people who choose distinct decision options in the game equilibrium.

According to this framework, we use the terms *x* and *x*′ for group A to denote individuals who use integrated versus nonintegrated strategies and *s*_*t*_(*x*) and *s*_*t*_(*x*′) to denote the proportion of individuals who use strategies x and x′ in group A at stage *t*, respectively. For group B, we define similar variables, *y* and *y*′ to denote individuals who use integrated versus nonintegrated strategies, and *s*_*t*_(*y*) and *s*_*t*_(*y*′) to denote the proportion of individuals who use strategies *y* and *y*′ in group B at stage *t*, respectively. Based on the above settings, we can then define the expected payoff functions for strategies *x* and *x*′, denoted as *u*_*t*_(*x*) and *u*_*t*_(*x*′), respectively, as shown in (1) and (2). The average expected payoff $\bar{u_{t}^{b}}$ for group A is shown in (3).

(1) $$\begin{array}{c} u_{t}\left(x\right)=s_{t}\left(y\right)\pi_{A}^{1}+s_{t}\left(y^{\prime }\right)\pi_{A}^{2}, \end{array}$$

(2) $$\begin{array}{c} u_{t}\left(x^{\prime }\right)=s_{t}\left(y\right)\pi_{A}^{3}+s_{t}\left(y^{\prime }\right)\pi_{A}^{4}, \end{array}$$

(3) $$\begin{array}{c} \bar{u_{t}^{b}}\;=s_{t}\left(x\right)u_{t}\left(x\right)+s_{t}\left(x^{\prime }\right)u_{t}\left(x^{\prime }\right). \end{array}$$

Based on the fundamental concept of Taylor and Jonker's replication dynamic (RD) model [18, 19], we can then derive the RD equations for firm A and firm B to choose an integration strategy, as illustrated in (4) and (5) They will be used in the next sections to conduct an analysis of the evolutionary game's stable strategy.

(4) $$\begin{array}{c} {\dot{s}}_{x}=s\left(x\right)\left[1-s\left(x\right)\right]\left[S_{A}-C_{A}+E_{A}+s\left(y\right)\left(L_{A}-E_{A}\right)\right., \end{array}$$

(5) $$\begin{array}{c} {\dot{s}}_{y}=s\left(y\right)\left[1-s\left(y\right)\right]\left[S_{B}-C_{B}+E_{B}+s\left(y\right)\left(L_{B}-E_{B}\right).\right. \end{array}$$

## 4. ESS Analysis

### 4.1. Parameter Discussion

An evolutionary stable strategy (ESS) is one that is formed when all individuals in a finite-information repeated game adjust their strategies continuously until they reach equilibrium. An ESS can be either static or changing in a cyclical fashion. We can discuss ESS with the help of RD equations [20, 21].

#### 4.1.1. Analysis for Firm A

Based on the RD equation of firm A, let *f*(*y*)=*a*_1_*s*(*y*)+*b*_1_, *a*_1_=*L*_*A*_ − *E*_*A*_, and *b*_1_=*S*_*A*_ − *C*_*A*_+*E*_*A*_. Then, (4) can be replaced by ${\dot{s}}_{x}=s\left(x\right)\left[1-s\left(x\right)\right]f\left(y\right)$, *s*(*x*) ∈ (0,1).

If *a*_1_=0, then the value of f(*y*) depends on the value of *b*_1_. If *b*_1_ > 0, then ${\dot{s}}_{x}>0$, and if *b*_1_ < 0 then ${\dot{s}}_{x}<0$.

If *a*_1_ ≠ 0, as *s*(*x*) ∈ [0,1], the value of *f*(*y*) depends on the value of −*b*_1_/*a*_1_. Hence, the value of −*b*_1_/*a*_1_ needs to be discussed under different conditions.

1. When −*b*_1_/*a*_1_ ≤ 0, if *a*_1_ > 0, then $\dot{s_{x}}>0$; if *a*_1_ < 0, then $\dot{s_{x}}<0$.
2. When 0 < −*b*_1_/*a*_1_ < 1, if *a*_1_ > 0 and −*b*_1_/*a*_1_ < *s*(*y*) ≤ 1, then $\dot{s_{x}}>0$, if *a*_1_ > 0 and 0 ≤ *s*(*y*) < −*b*_1_/*a*_1_, then $\dot{s_{x}}<0$, if *a*_1_ < 0 and 0 ≤ *s*(*y*) < −*b*_1_/*a*_1_, then $\dot{s_{x}}>0$, if *a*_1_ < 0, and −*b*_1_/*a*_1_ < *s*(*y*) ≤ 1, then $\dot{s_{x}}<0$, and if *s*(*y*)=−*b*_1_/*a*_1_, then $\dot{s_{x}}=0$.
3. When −*b*_1_/*a*_1_ ≥ 1, if *a*_1_ > 0, then $\dot{s_{x}}<0$; if *a*_1_ < 0, then $\dot{s_{x}}>0$.

Through the above discussion, we can conclude that if −*b*_1_/*a*_1_ ≤ 0 or −*b*_1_/*a*_1_ ≥ 1, the value of $\dot{s_{x}}$ is not affected by the value of *s*(*y*), which means that, under this condition, firm A's decision is not affected by the choice of firm B. Otherwise, if 0 < −*b*_1_/*a*_1_ < 1, firm A's decision is affected by the choice of firm B.

#### 4.1.2. Analysis for Firm B

Based on the RD equation of firm B, let *g*(*x*)=*a*_2_*s*(*x*)+*b*_2_, *a*_2_=*L*_*B*_ − *E*_*B*_, and *b*_2_=*S*_*B*_ − *C*_*B*_+*E*_*B*_; then, $\dot{s_{y}}=s\left(y\right)\left[1-s\left(y\right)\right]g\left(x\right)$. Similarly, we can conclude that if −*b*_2_/*a*_2_ ≤ 0 or −*b*_2_/*a*_2_ ≥ 1, the value of $\dot{s_{y}}$ is not affected by the value of *s*(*x*), which means that firm B's decision is not affected by the choice of firm A under this condition.

However, if 0 < −*b*_2_/*a*_2_ < 1, firm B's decision will depend on the action of firm A. Different situations under different parameter values are shown in Table 2.

According to the results of the preceding analysis (as shown in Table 2), there are three basic game relationships: unrelated, one-way influence, and mutual influence. Each of these three scenarios will be discussed further below.

### 4.2. RD Process Analysis for the Unrelated Situation

In such states, the decisions of firms A and B do not affect each other. For example, if −*b*_1_/*a*_1_ ≤ 0, *a*_1_ < 0, −*b*_2_/*a*_2_ ≥ 1, and *a*_2_ > 0, then $\dot{s_{x}}<0$ and $\dot{s_{y}}<0$. At this stage, as illustrated in Figure 3, the average probability that firms A and B will choose an integration approach diminishes, resulting in an ESS of (nonintegration, nonintegration). Similarly, we can derive more ESSs for this condition, as detailed in Table 3.

### 4.3. RD Process Analysis under One-Way Influence

This situation can be further classified into two categories based on the variations in the game's dominant player: (1) the one-way influence game in which firm A exerts influence over firm B and (2) the one-way influence game in which firm B exerts influence over firm A. For example, if *s*(*y*) ∈ [0, −*b*_1_/*a*_1_), −*b*_1_/*a*_1_ ∈ (0,1),  *a*_1_ > 0, −*b*_2_/*a*_2_ ≤ 0, and *a*_2_ > 0, then $\dot{s_{y}}>0$; if *s*(*y*) ∈ [−*b*_1_/*a*_1_, 1), −*b*_1_/*a*_1_ ∈ (0,1), *a*_1_ > 0, −*b*_2_/*a*_2_ ≤ 0 and *a*_2_ > 0, then $\dot{s_{x}}>0$. The RD process is shown in Figure 4.

The preceding results imply that if firm B's initial likelihood of integrating is within [0, −*b*_1_/*a*_1_), firm B is more likely to select the integration strategy. When this likelihood reaches the interval [−*b*_1_/*a*_1_, 1), firm B's decision begins to impact firm A, favoring the integration option. This step is repeated until the strategy's final ESS for both is established (integration, integration). Additional ESS results in this state are listed in Table 4.

### 4.4. RD Process Analysis in the Mutual Affect Situation

When −*b*_1_/*a*_1_ ∈ (0,1) and −*b*_2_/*a*_2_ ∈ (0,1), the decisions of firms A and B mutually affect each other.

When *a*_1_*a*_2_ > 0, if *s*(*y*) ∈ [0, −*b*_1_/*a*_1_), −*b*_1_/*a*_1_ ∈ (0,1), *a*_1_ < 0, −*b*_2_/*a*_2_ ∈ (0,1)  and *a*_2_ < 0, then $\dot{s_{x}}>0$; if *s*(*y*) ∈ [−*b*_1_/*a*_1_, 1), −*b*_1_/*a*_1_ ∈ (0,1), *a*_1_ < 0, −*b*_2_/*a*_2_ ∈ (0,1)  and *a*_2_ < 0, then $\dot{s_{x}}<0$; if *s*(*x*) ∈ [0, −*b*_2_/*a*_2_), −*b*_1_/*a*_1_ ∈ (0,1), *a*_1_ < 0, −*b*_2_/*a*_2_ ∈ (0,1) and *a*_2_ < 0, then $\dot{s_{y}}>0$; and if *s*(*x*) ∈ [−*b*_2_/*a*_2_, 1), −*b*_1_/*a*_1_ ∈ (0,1), *a*_1_ < 0, −*b*_2_/*a*_2_ ∈ (0,1)  and *a*_2_ < 0, then $\dot{s_{y}}<0$. The RD process for the preceding situation is depicted in Figure 5, and the figure contains four sections, A–D. If (*s*(*x*),  *s*(*y*)) is located in region A, then ESS is (nonintegration, integration), which means that firm A pursues a nonintegration strategy, whereas firm B pursues an integration strategy. If (*s*(*x*),  *s*(*y*)) is located in region C, then ESS is (nonintegration, integration). If (*s*(*x*),  *s*(*y*)) is located in region B or D, then ESS is (integration, nonintegration) or (nonintegration, integration). When 0 < −*b*_1_/*a*_1_ < 1, *a*_1_ > 0 and 0 < −*b*_2_/*a*_2_ < 1, *a*_2_ > 0, see Table 5 for the relevant results.

When *a*_1_*a*_2_ < 0, if *s*(*y*) ∈ [−*b*_1_/*a*_1_, 1), −*b*_1_/*a*_1_ ∈ (0,1),  *a*_1_ > 0, −*b*_2_/*a*_2_ ∈ (0,1) and *a*_2_ < 0, then $\dot{s_{x}}>0$; if *s*(*y*) ∈ [0, −*b*_1_/*a*_1_), −*b*_1_/*a*_1_ ∈ (0,1), *a*_1_ > 0, −*b*_2_/*a*_2_ ∈ (0,1) and *a*_2_ < 0, then $\dot{s_{x}}<0$; if *s*(*x*) ∈ [0, −*b*_2_/*a*_2_), −*b*_1_/*a*_1_ ∈ (0,1), *a*_1_ > 0, −*b*_2_/*a*_2_ ∈ (0,1) and *a*_2_ < 0, then $\dot{s_{y}}>0$; and if *s*(*x*) ∈ [−*b*_2_/*a*_2_, 1), −*b*_1_/*a*_1_ ∈ (0,1), *a*_1_ > 0, −*b*_2_/*a*_2_ ∈ (0,1), and *a*_2_ < 0, then $\dot{s_{y}}<0$. The RD process is shown in Figure 6. Finally, there is only one stable state in which each side will adapt to the mixed strategy and the ESS is (−*b*_2_/*a*_2_, −*b*_1_/*a*_1_). Similarly, when −*b*_1_/*a*_1_ ∈ (0,1), *a*_1_ < 0 and −*b*_2_/*a*_2_ ∈ (0,1), *a*_2_ > 0, we obtain the results shown in Table 5.

## 5. Case Study

### 5.1. Background

The iron ore trade value between Australia and China is growing rapidly. According to the latest data from the China Iron and Steel Association (CISA), the volume of Chinese iron ore imports from Australia in 2020 was 713 million tons (accounting for 60.9% of the year's total). Western Australia is the main producer of iron ore in Australia, accounting for 99% of Australia's iron ore production. Western Australia had 836 Mt of iron ore sales in 2019–2020, which were mostly exported to China (83 percent). The main origin in Western Australia is the Pilbara Region (accounting for 97%), as shown in Figure 7.

According to the data from the Government of Western Australia Department of Mines and Petroleum, there are approximately 17 principal iron ore producers in Western Australia. Among them, three companies, Rio Tinto, BHP Billiton, and Fortescue Metals Group, account for more than 90% of production. These companies have built their own export supply chains, including rail lines and port facilities, as shown in Table 6.

Thus far, through joint-venture packages, which include Chinese firms taking minority equity stakes and offering long-term contracts for new iron ore exports, many Chinese steel-producing firms have taken measures to integrate their supply chains, as shown in Table 7.

### 5.2. Numerical Examples

We designed different scenarios based on data collected from Chinese steel-producing companies and iron-ore suppliers in Australia to analyze the best options for Chinese steel-producing firms. We observe two primary patterns used in SCI: the joint-venture pattern (which includes long-term contracts) and the self-support pattern. Figures 8 and 9 depict two integrated supply chain patterns. As a result, we created two cases, one to represent each integration pattern.

As firms with different market scales have different cost structures, we need to consider the influence that market scale has on decision-making. We choose Baosteel Group and Benxi Steel as targets, which are Chinese steel-producing firms but do not have same level of production. According to the data from the World Steel Association, their crude steel production for the period 2017–2020 is listed in Table 8. We chose their net profits in 2011 as original profits, which were US$ 2.895 billion and US$542 million. Therefore, their unit profits in 2011 were US$ 66.8/ton and US$ 32.8/ton. Hence, *P*_*A*_=66.8 and *P*_*B*_=32.8. Following that, we will consider two scenarios. In scenario 1, we assume that both players can only use the “joint-venture pattern” to integrate their supply chains. We suppose in scenario 2 that they can only follow the “self-support pattern.”

#### 5.2.1. Scenario 1

In scenario 1, we consider the joint-venture pattern. Under this condition, Chinese steel-producing firms obtain cheaper iron ore by taking minority equity stakes and offering long-term contracts for new iron ore exports. As most Chinese steel-producing companies are in the process of integration projects, it is difficult to calculate supply chain cost savings from the whole raw material cost. Therefore, we obtain data on supply chain cost savings from iron ore producers in Australia, which provided the cost savings from integrating their export supply chains in their annual reports. Take, for example, the case of FMG, which committed to expansion in November 2010. We chose its cost data after expansion. As in the previous discussion, we believe that the supply chain cost saving consists of the saving of rail costs, port costs, and shipping costs. By decreasing the average cost, we can obtain *S*_*A*_=3.6, *S*_*B*_=3.6.  Table 9.

To determine the cost of SCI in this model, we choose two real cases. One is Baosteel Group's investment in Aquila in 2009. In this case, Baosteel Group invested as much as US$285.6 million in Aquila to obtain a 50% share of one 30 Mtpa project. The other case is Shougang investment in Balmoral in 2008. The specific data are shown in the table below. Assuming that the costs are shared equally from 2011 to 2014, we can obtain *C*_*A*_=1.65 and *C*_*B*_=1.04.

As the steel-producing market is oligopolistic, we assume that company A with a larger market share will gain 10% excess profits if only it implements the SCI strategy. Otherwise, it will face a 20% excess loss. The same situation for company B (smaller market share) is 20% excess profits and 10% excess loss. Therefore, we can obtain *E*_*A*_=6.68, *L*_*A*_=13.36, *E*_*B*_=6.56, and *L*_*B*_=3.28. By applying MATLAB, we obtain the ESS (integration, integration) after deriving hundreds of initial solutions, as shown in Figure 10.

It means that in the short term, firms A and B will choose the joint-venture pattern for SCI. We perform a sensitivity analysis on the proportional coefficient of fixed asset investment loss *P*. The calculation shows that the ESS is (integration, integration) for any *P*. It indicates that the decisions of firms A and B are not affected by the coefficient *P* in the short term if they are integrated using the joint-venture pattern.

#### 5.2.2. Scenario 2

In Scenario 2, we consider the self-support model. The data on original profits are the same. Hence, *P*_*A*_=66.8 and *P*_*B*_=32.8. We also obtain data on supply chain cost savings from the case of FMG. The total delivered cost of FMG was significantly lower in 2014 than in 2011, as shown in Table 10, because of its expansion in the supply chain. However, as a result of their small size and comparatively high costs, it is unlikely that most of these projects will be cost-competitive with the Big-3 incumbents. Therefore, we assume that *S*_*A*_=13.5 (15 ∗ 90%) and *S*_B_ = 12 (15 ∗ 80%).

We choose BHP exploration projects as the data source. These projects included the Jimblebar Mine Expansion project and Orebody 24 mine project. The Jimblebar Mine expansion project costed U.S.$3.6 billion and achieved a capacity of 35 Mtpa. The Orebody 24 mine project costed U.S.$0.7 billion and achieved a capacity of 17 Mtpa after one year of construction. Both projects were approved in 2011 and lasted 4 years. Then, we can obtain *C*_*A*_=24.28 and *C*_*B*_=16.12. Similar to Scenario 1, *E*_*A*_=6.68, *L*_*A*_=13.36, *E*_*B*_=6.56, and *L*_*B*_=3.28. By applying MATLAB, we obtain the ESS (0.74, 0.61) after conducting hundreds of initial solutions, as shown in Figure 11.

Additionally, we conduct a sensitivity analysis for *P* in the following section. We make *P* take values between 0 and 1 and perform the calculations, obtaining the following results.

When 0 ≤ p ≤ 0.106, the dynamic evolutionary process will reach an equilibrium state characterized by mixed strategies. As illustrated in Figure 12, the ESS equilibrium state moves to the upper left as the value of p increases, indicating that the probability of firm A (with a large market share) choosing an integration strategy continues to decrease, while the probability of firm B choosing an integration strategy increases. Note that because the investment loss ratio coefficient *P* can be interpreted as the probability of experiencing policy risk, the results of this calculation indicate that the probability of choosing an integration strategy for firm a with its dominant market share decreases significantly as the probability of experiencing policy risk increases.

When 0.106 < p ≤ 0.151, −b1/*a*1 ≥ 1, and 0 < –b2/*a*2 < 1. It means that in this case, the strategy evolution process of firm A is not influenced by the decision of firm B, while the strategy evolution process of firm B is influenced by firm A. In this case, the ESS is (nonintegration, integration), i.e., firm A chooses not to integrate, and firm B chooses to integrate. It indicates that as the probability of policy risk expands further, firm A's decision will change from preferring integration to nonintegration, while firm B still prefers to choose integration.

When p > 0.151, −*b*_1_/*a*_1_ ≥ 1, and −*b*_2_/*a*_2_ ≤ 0. Here, the strategy evolution processes of firms A and B are independent. At this stage, the ESS is (nonintegration, nonintegration). This finding implies that when risk reaches a particular level, both types of firms choose to pursue a nonintegration strategy. This outcome is entirely consistent with our expectations.

### 5.3. Discussion

The findings of the preceding study are congruent with the reality of the situation. Actual economic and trade data indicate that the relationship between China and Australia has a substantial impact on investment activity between the two countries. Because of ongoing tensions between the two nations, Chinese investment in Australia fell to its lowest level in nearly six years in 2020, as shown in Figure 13, by 61% year-on-year to $783 million from $2.08 billion the previous year. There were only 20 Chinese investment projects in Australia throughout 2019, far fewer than the 111 in 2016. From the standpoint of steel SCI, the model described in this article provides a quantitative explanation for this phenomenon.

In Scenario 1, the value of each parameter accords with the situation “unrelated,” which means that firms A and B will make decisions based on their own situations, without considering the competitor's strategy. In this case, both of them will gain profits if they apply an SCI strategy. Additionally, we can see that, regardless of the value of *p*, neither side of the game can affect the other's decisions in Scenario 1, and the ESS is (integration, integration). It is primarily because both parties to the game employ the short-term joint venture pattern for SCI, which is an “asset-light pattern” with low investment and risk, and thus the integration decision effectively mitigates political concerns.

Unlike in Scenario 1, we assume that both players adopt the self-support pattern for SCI in Scenario 2. Because this model requires significant investment and is essentially a fixed asset investment, it can be considered an “asset-heavy pattern.” While SCI based on the self-support pattern can significantly reduce operating costs and increase efficiency, there is a significant investment risk associated with it. If the countries' relationship deteriorates, it will result in a series of irreversible and significant losses for the firms.

Note that the political risk factor has varying effects on firms in various market positions under the self-support pattern. Specifically, as risk (p) increases, the probability that firm A will choose the integration strategy decreases continuously until *p*=0.106, at which point firm A becomes unwilling to choose the integration strategy, however, firm B always prefers the integration strategy when p is less than 0.106. At *p*=0.151, the response of firm B changes. It demonstrates that even when p is less than 0.151, firm B is willing to accept the risk posed by policy factors. When p exceeds 0.151, firm B is also forced to abandon its integration strategy because of the high policy risk.

## 6. Summary and Conclusions

In this paper, we developed an evolutionary game model to analyze the decision-making of an SCI strategy for steel-producing firms. Considering the characteristics of an oligopolistic market, we formulated the supply chain decision-making problem as an asymmetric RD model and then proposed an RD process analysis to obtain every ESS result under different parameter situations. In addition, two scenarios were designed to demonstrate that such problems can be formulated and solved well by an evolutionary game model. Importantly, this paper adds to the literature by empirically testing the SCI strategy indirectly. Furthermore, it also allows for the generalization of special cases of oligopolistic market equilibrium problems and provides a detailed case study of Chinese steel-producing firms' iron ore supply chain.

In conclusion, there are some limitations of the research in this paper that suggest that future studies can be extended in several directions. Firstly, the complexity of participators' behavior in this oligopolistic market has been simplified in this evolutionary game model. Future studies can consider the cost structure of steel-producing firms and introduce a pricing model to analyze the extra profits and losses that each firm may face. Secondly, collecting data from steel-producing firms' supply chains could be more appropriate for evaluating the cost savings of the total supply network. Therefore, future research should replicate and integrate our study using numerical data from iron ore-producing firms. Obviously, it would also be worthwhile for further theoretical developments and empirical applications.

## Figures and Tables

**Figure 1:** Comparison of cumulative annual data of Australian iron ore imports, 2006–2020.

**Figure 2:** The four situations of the game.

**Figure 3:** The evolutionary process in the unrelated situation.

**Figure 4:** The evolutionary process of one-way influence.

**Figure 5:** The evolutionary process of mutual effect under *a*_1_*a*_2_ > 0.

**Figure 6:** The evolutionary process of mutual effect under *a*_1_*a*_2_ < 0.

**Figure 7:** Iron ore transport routes between Australia and China.

**Figure 8:** Joint-venture mode.

**Figure 9:** Self-support model.

**Figure 10:** The simulation result of Scenario 1.

**Figure 11:** The simulation result of Scenario 2.

**Figure 12:** The comparison of simulation results under *p*=0 & *p*=0.09.

**Figure 13:** China's investment in Australia 2015–2020 ($ billion).

**Table 1:** The payoff under different situations.

Firms A	Firms B	
	Integration	Nonintegration
Integration	(*P*_*A*_+*S*_*A*_ − *C*_*A*_ − *R*_*A*_, *P*_*B*_+*S*_*B*_ − *C*_*B*_ − *R*_*B*_)	(*P*_*A*_+*S*_*A*_ − *C*_*A*_ − *R*_*A*_+*E*_*A*_, *P*_*B*_ − *L*_*B*_)
Nonintegration	(*P*_*A*_ − *L*_*A*_, *P*_*B*_+*S*_*B*_ − *C*_*B*_ − *R*_*B*_+*E*_*B*_)	(*P*_*A*_, *P*_*B*_)

where *P*_*A*_,  *P*_*B*_ are the original profits of group A and group B under the nonintegration strategy. *S*_*A*_,  *S*_*B*_ are the supply chain cost savings of group A and group B under the integration strategy. *C*_*A*_,  *C*_*B*_ are the costs of supply chain integration of group A and group B. *R*_*A*_,  *R*_*B*_ are the SCI costs of risk *R*_*A*_ = *αC*_*A*_, *R*_B_ = *αC*_B_, where *α* is the investment loss ratio. *E*_*A*_,  *E*_*B*_ are the extra earnings of group A and group B. *L*_*A*_,  *L*_*B*_ are the extra losses of group A and group B.

**Table 2:** Game situations under different parameter values.

Classification	Situation	Parameter values of firm A	Parameter values of firm B
Unrelated	Firms A and B are independent of each other	*a*_1_=0 or −*b*_1_/*a*_1_ ≤ 0 or −*b*_1_/*a*_1_ ≥ 1	*a*_2_=0 or −*b*_2_/*a*_2_ ≤ 0 or −*b*_2_/*a*_2_ ≥ 1
One-way influence	Firm B is affected by firm A	*a*_1_=0 or −*b*_1_/*a*_1_ ≤ 0 or −*b*_1_/*a*_1_ ≥ 1	0 < −*b*_2_/*a*_2_ < 1
	Firm A is affected by firm B	0 < −*b*_1_/*a*_1_ < 1	*a*_2_=0 or −*b*_2_/*a*_2_ ≤ 0 or −*b*_2_/*a*_2_ ≥ 1
Mutual influence	Firms A and B interact with each other	0 < −*b*_1_/*a*_1_ < 1	0 < −*b*_2_/*a*_2_ < 1

**Table 3:** ESS in the unrelated situation.

Classification	Parameter value of firm A	ESS	Parameter value of firm B	ESS

Unrelated	−*b*_1_/*a*_1_ ≤ 0 and *a*_1_ < 0	0	−*b*_2_/*a*_2_ ≤ 0 and *a*_2_ < 0	0
	−*b*_1_/*a*_1_ ≤ 0 and *a*_1_ > 0	1	−*b*_2_/*a*_2_ ≤ 0 and *a*_2_ > 0	1
	−*b*_1_/*a*_1_ ≥ 1 and *a*_1_ < 0	1	−*b*_2_/*a*_2_ ≥ 1 and *a*_2_ < 0	1
	−*b*_1_/*a*_1_ ≥ 1 and *a*_1_ > 0	0	−*b*_2_/*a*_2_ ≥ 1 and *a*_2_ > 0	0

**Table 4:** ESS in the situation that only one party is affected.

Classification	Parameter value of firm A	Parameter value of firm B	ESS

Firm B influences firm A	0 < −*b*_1_/*a*_1_ < 1 and *a*_1_ > 0	−*b*_2_/*a*_2_ ≤ 0 and *a*_2_ < 0	(0, 0)
		−*b*_2_/*a*_2_ ≤ 0 and *a*_2_ > 0	(1, 1)
		−*b*_2_/*a*_2_ ≥ 1 and *a*_2_ < 0	(1, 1)
		−*b*_2_/*a*_2_ ≥ 1 and *a*_2_ > 0	(0, 0)
	0 < −*b*_1_/*a*_1_ < 1 and *a*_1_ < 0	−*b*_2_/*a*_2_ ≤ 0 and *a*_2_ < 0	(1, 0)
		−*b*_2_/*a*_2_ ≤ 0 and *a*_2_ > 0	(0, 1)
		−*b*_2_/*a*_2_ ≥ 1 and *a*_2_ < 0	(0, 1)
		−*b*_2_/*a*_2_ ≥ 1 and *a*_2_ > 0	(1, 0)

Firm A influences firm B	−*b*_!_/*a*_1_ ≤ 0 and *a*_1_ < 0	0< −*b*_2_/*a*_2_ < 1 and *a*_2_ > 0	(0, 0)
	−*b*_1_/*a*_1_ ≤ 0 and *a*_1_ > 0		(1, 1)
	−*b*_1_/*a*_1_ ≥ 1 and *a*_1_ < 0		(1, 1)
	−*b*_1_/*a*_1_ ≥ 1 and *a*_1_ > 0		(0, 0)
	−*b*_1_/*a*_1_ ≤ 0 and *a*_1_ < 0	0< −*b*_2_/*a*_2_ < 1 and *a*_2_ < 0	(1, 0)
	−*b*_1_/*a*_1_ ≤ 0 and *a*_1_ > 0		(0, 1)
	−*b*_1_/*a*_1_ ≥ 1 and *a*_1_ < 0		(0, 1)
	−*b*_1_/*a*_1_ ≥ 1 and *a*_1_ > 0		(1, 0)

**Table 5:** ESS under mutual influence.

Situations	Parameter of firm A	Parameter of firm B	ESS

Mutual influence	0 < −*b*_1_/*a*_1_ < 1 and *a*_1_ < 0	0< −*b*_2_/*a*_2_ < 1 and *a*_2_ < 0	(0, 1) or (1, 0)
	0 < −*b*_1_/*a*_1_ < 1 and *a*_1_ > 0	0< −*b*_2_/*a*_2_ < 1 and *a*_2_ > 0	(0, 0) or (1, 1)
	0 < −*b*_1_/*a*_1_ < 1 and *a*_1_ > 0	0< −*b*_2_/*a*_2_ < 1 and *a*_2_ < 0	(−*b*_2_/*a*_2_, −*b*_1_/*a*_1_)
	0 < −*b*_1_/*a*_1_ < 1 and *a*_1_ < 0	0< −*b*_2_/*a*_2_ < 1 and *a*_2_ > 0	(−*b*_2_/*a*_2_, −*b*_1_/*a*_1_)

**Table 6:** Iron ore export supply chain of the main producers.

Iron ore producer	Rail (km)	Port facility

Rio Tinto	1600	4 ports with 11 berths (Dampier port)
BHP	1000	8 berths (port Hedland)
FMG	620	4 berths and 1 under construction (port Hedland)

**Table 7:** Investment of Chinese steel-producing firms.

Firm	Project	Value (A$ millions)	Size (Mtpa) and associated LTCs (% of output)

Ansteel	Karara JV	530	Plan 10 (100%)
Shougang	Balmoral south	58	Plan 12 (100%)
Shagang	Grange	NA	2.5 (100%)
Baosteel	Aquila	286	Plan 30 (50%)

**Table 8:** Crude steel production, 2017–2020.

Tonnage (million tonnes)	2017	2018	2019	2020
Baosteel group	46.17	47.10	46.88	45.62
Benxi steel	15.49	15.47	15.83	16.63

**Table 9:** FMG supply chain cost after expansion.

Supply chain costs U.S.$ m	After 1 year	After 2 years	After 3 years	After 4 years

Rail costs	128	139	182	238
Port costs	97	125	181	252
Shipping cost	509	672	769	1210
Ore shipped	40.9	57.5	75.9	118.4
Average cost U.S.$/wmt	17.95	16.28	14.91	14.35

**Table 10:** Total delivered cost of FMG.

Supply chain costs	2011	2012	2013	2014

Total delivered cost US$/wmt	67	69	62	52

## Data Availability

No data were used to support this study.
